The article "Analysis of the Implementation Effect of College Curriculum Ideological and Political under the Background of Ecological Sustainable Development" was retracted in 2023. Reasons: unreliable results or conclusions; concerns about the data; concerns about the peer review; concerns about the citations.

# Analysis of the Implementation Effect of College Curriculum Ideological and Political under the Background of Ecological Sustainable Development

**DOI:** 10.1155/2022/3937168

**Published:** 2022-08-09

**Authors:** Xiaoli Wu, Dang Wu, Xiufeng Ma

**Affiliations:** ^1^School of Marxism, Handan University, Handan 056000, China; ^2^School of Special Education, Handan University, Handan 056000, China; ^3^School of Economics and Management, Handan University, Handan 056000, China

## Abstract

Our country is paying more and more attention to ecological issues. How to put ecological sustainable development in real life is a key problem. This article discusses the significance of integrating ecological sustainable development and college ideological political courses. Therefore, an experiment was designed to analyse the model of ecology and other courses. The final experiment showed the following: (1) The ecological sustainable development model can be well integrated into the students in their courses. Students can freely choose to study some quality assurance thought courses and reinforce their spiritual level. The mentality of this model can also self-optimize to solve students' troubles in choosing courses and consider the level of students intimately. (2) According to the experimental data of the figures and tables, it is concluded that the form “other professional courses” at my country is still very serious, and the popularization of ideological and political courses is not common, so it is a little troublesome to carry out work, but our system model is very characteristic. With its help, we have obtained the effect of the integration of ecological sustainable development and students' curriculum. The state has vigorously provided economic support for their development. Under their influence, students have gradually maintained their awareness of protecting the environment. Socioeconomic and environmental conditions are also improving. However, in the future, the times will change, and we will continue to update the system model to adapt to more challenges.

## 1. Introduction

Ecological environment describes the role of IS in ecological sustainable development and raises three issues of ecological efficiency, ecological fairness, and ecological benefit. We put many things of ecological sustainable development into this system to achieve more approach to environmental ecology, underscoring the importance of practitioners in understanding the environmental impacts of IS development or use, and the role IS plays in promoting large-scale research on environmental sustainability [1]. This paper describes the impact of the soil ecological environment of Kembela Village, West Kalimantan, Indonesia, and investigates the content of microcomponents, such as pH and phosphorus molecules, in the cultivated soil from decades ago to present, and infers that the ecological environment of the land after cremation is better. This development model is sustainable development [2]. A potential reconciliation theory for exploring environmental sustainability and individual well-being is mentioned in Ecological Sustainability, and analysis of related theoretical and empirical evidence suggests that environmental degradation makes it difficult to meet the needs for security, capacity, connectivity, and autonomy; there is now a need for sustainable development that meets these four needs to improve the situation. These include shifting values from external, materialistic goals to internal goals to help people choose a more ecologically sustainable way of life [3]. It describes the issues of sustainable development and environmental protection discussed by the United Nations. The sustainable development of the Arab world is facing major dangers. The living environment of human beings is developing in positive and negative directions. According to the current data, in order to discuss the most important demographics and sustain the development path of the Arab countries, we propose partial ecological integration based on exchange of vegetables, items, and coolies, which is the greatest hope for improving Arab restoration and sustainable development [4]. Sustainable development has always been center information for ecological protection and state regulations, but that understanding landscape and sustainability issues leaves much to be desired. The spatial land use uninterrupted index project aims to improve spatially unique metrics for mapping environmental uninterrupted. Environmental sustainability is defined in terms of uncertainty and environmental complexity and is used to assess environmental sustainability, which can show similar results despite differences in these methods. Landscape structure indicators have been the reason why they are the standard by which a good ecological environment can develop uninterruptedly; that is, they are connected with the ecological environment features of the landscape [5]. Over time, the environment needs to be addressed through the spatial scales associated with higher land use, from a single farmer's farm to the rest of the world. In addition to the production efficiency and sustainability of agroecosystems, as an important factor in sustainable development, the speed with which production patterns recover from deterioration. Consider temporal and spatial projections of processes affecting sustainability, in particular the movement of energy, wind, water, and nutrients, as well as climate change and natural disasters [6]. Ideological teaching to students is the fundamental requirement of education, which not only includes unique Chinese traditional thinking, but also includes the reform of educational concepts in the rapidly changing new era. It is very common and has gained some applied educational methods at colleges and universities, but in some areas, there is still room for improvement. It is an important part of classroom teaching for college teachers to implement good ideas. Therefore, college teachers should do everything possible to deepen the connotation and meaning of thoughts, understand the specific issues of ideology and politics, focus on development of courses and the main methods of classrooms, and apply practical theories and courses [7]. “Course Ideology and Politics” is a new educational concept that combines personal ideological teaching with politics. With the development of our country, the application of foreign language skills is in very high demand. As a course that combines cross-cultural knowledge with the purity of foreign cultural systems, college English courses must meet the great demand of college students for ideological and political ideas that change the content and methods of teaching. Change college English teaching, go beyond traditional English teaching, deepen the transformation of translation teaching, and cultivate intercultural communication skills and modern applications of higher academic education forecasting [8]. Ideological and political learning can be explained in other ways. Based on this problem, we revise the curriculum and improve the teaching plan, teaching methods, and assessment methods in the curriculum. Throughout the course, we hope to enhance students' patriotism, stimulate their innovative thinking and entrepreneurial spirit, and ultimately cultivate a balanced attitude towards life, worldview, and values. Finally, make some contributions psychological education reform of college courses [9]. College curriculum ideology and politics is a creative conception to realize the core mission of Rieter to cultivate people. The same intellectual and political resources form a valuable coalition of leaders in the process of knowledge transfer and skill development, helping students affirm their values and beliefs, and foster patriotism and personal education. Therefore, teachers should not only provide technical skills, but also start from the basis of “education,” emphasize the ideological and political issues of character teaching, and attach importance to the value management of organic relationships. The application of ideology and politics in the study of construction drawings in colleges is discussed, and then the steps for incorporating ideological and political elements into learning materials to provide teaching guidance are highlighted [10]. With the steady upward of network technology today, the courses of online colleges and universities are becoming more and more popular. In fact, the platform a network of them and services provided by social networks. Given the enormous value of the Internet in community and community education, we need to fully recognize the new opportunities and challenges brought about by the rapid development of the Internet in traditional and community education and make existing systems useable. Ideological education community education, political science ideology, and political network: how to use online services effectively in academic; how to work effectively in social networks through academic and political education; how to strengthen teaching system; and how do websites understand politics and policy? These are important questions that our current research at the university should answer [11]. Environmental values in ideological and political education are gradually emerging to better solve environmental and environmental problems. On the one hand, we need to understand what it means, and on the other hand, we must consider the principles outlined in Marx's book of the environment. It is also important to discuss and assess environmental values in relation to ideas and policies that threaten society in different ways [12]. The current university teaching concept is based on the “online and offline” teaching system. In my country's education system, ideology and politics are closely related to educational goals. The contemporary teaching concept is mainly to combine ideological and political courses with daily learning, that is, on the basis of “online and offline integration.” This time, a university English language course is used to discuss the relationship between blended learning and ideological and political learning, to explore blended teaching methods, and to make suggestions on how to restructure the assessment system to provide information [13]. With the rapid development of my country's education field, the integration of network technology and schools is bound to evolutionary trend. In the context of the Internet, they are also in full swing. In the process of development, we should improve and innovate, analyze the new development path of the Internet, and improve the quality of the new school reform through innovative development. It is necessary to pay attention to continuity of excellent previous ecological concept and to realizing the biological connection between the Internet and ideology and politics [14]. Curriculum-based ideology is at the center of educational research and reform. According to the initial literature collection of the knowledge database, the use of time allocation, survey sources, research authors, and so on to analyse keywords, and so on, it is found that there are still many problems in ideology and politics, and we still need continuous efforts to change this phenomenon [15].

The article "Analysis of the Implementation Effect of College Curriculum Ideological and Political under the Background of Ecological Sustainable Development" was retracted in 2023. Reasons: unreliable results or conclusions; concerns about the data; concerns about the peer review; concerns about the citations.

## 2. Ecological Sustainable Development Analysis

### 2.1. Definition of Ecological Sustainability

Ecologically sustainable development is development that responds to contemporary needs without compromising the latter; it should have the ability to apply this phenomenon to its own needs. They form a together provision that requires not only the purpose of socioeconomic growth, but also the protection of many ecological environments they use (e.g., freshwater, ocean, etc.). The focus of sustainable development is economic and social development, strong social governance, and the improvement of human quality; always developing utilization of resources is a necessary condition for the sustainable development of the world. People are the focus of sustainable development. Sustainability is real progress.

### 2.2. Principles of Ecological Sustainability

Fairness principle: Intergenerational equality, resource allocation, and use equality. Ecological sustainable development is an opportunity and an advantage. It also strikes the balance between generations and regions, in other words, to be able to guarantee the current requirements without disturbing future. The principle of generational productivity proves that all generations live in a and have the same right to life. To this end, ecological sustainable development makes poverty eradication. There is a major problem that needs to be solved in all countries and regions. Sustainability principle: In other words, there must be constraints to meet demand; the concept of development contains constraints; the word “evolution” also contains constraints. Therefore, environment, resources, and social engineering and organizational conditions limit the environment's ability to meet current needs. The most serious condition is the infrastructure it depends on: natural objects and ecological protection. It can be seen that sustainable performance links the real interests of people with the real interests of the people. The principle of universality: Although ecological models in different countries will be different, it is common to develop the principles of equality. The integrity and connectedness of the planet dictates that the planet must come together to recognize our home. Ecological sustainability analyzes international issues through cultural and historical barriers. The problems addressed there involve everyone, that is internal affairs and foreign affairs, and the common goal of sustainable development can only be achieved through the joint efforts of all parties and the combination of people's individual interests and common interests.

The article "Analysis of the Implementation Effect of College Curriculum Ideological and Political under the Background of Ecological Sustainable Development" was retracted in 2023. Reasons: unreliable results or conclusions; concerns about the data; concerns about the peer review; concerns about the citations.

### 2.3. The Basic Connotation of Ecological Sustainable Development

In 2002, my country took the uninterrupted development of the ecological environment as the main goal, which can ensure economic growth and change people's current way of life, which will gradually become a new society, ethics and civilization, and its basic connotations are as follows: Pay attention to development issues. Growth is different from economic upturn, growth is a combination of social, technological, cultural, and many other phenomena. The sustainable development of the people, economic and social development shall not exceed the bearing capacity of natural; Fair exchanges between people, everyone today should strive to ensure that future generations develop and take advantage of the same development opportunities, and the development of a generation is the development of the few, not affecting the interests of others. The continuous coexistence of man and nature requires people to establish new values and limit; we must know how to care for nature, learn more about nature, and make progress together with nature. The sustainability of social development and economic development is the basic requirement of development. Make overall plans and take the road of civilization. The final decision, which is conducive to sustainable development, is an important historical milestone in the development of human civilization.

### 2.4. The Significance of Ecological Sustainability

At the beginning of the twenty-first century, the main goal of my country's sustainable development was to continuously improve the potential of sustainable development, achieve excellent results in economic restructuring, effectively control the entire population, and “significantly improve environmental conditions and increase resource utilization.” “It promotes the harmony between man and nature”. It helps the whole society to realize civilized production. The form of development includes the development of production, the prosperity of life and the good ecology. By adjusting the strategic structure of the national economy, we can optimize and upgrade the industrial structure, release resources and environment, change the balance of regional development, and narrow the gap between urban and rural areas.. Efforts are made to promote hunger eradication and poverty alleviation, continuously improve regional production and living conditions, strengthen infrastructure construction, improve the environment, and gradually transform the economic households that have not been lifted out of poverty to live a better life. Here are a few key points: Implement sustainable development policies to promote the combination of environmental benefits, economic benefits and social benefits. Promote the harmonious development of the economy, people, resources, and the environment, which is conducive to the transition of the economy from strong growth to strong growth, promotes sustainable, stable, and healthy economic development, and improves people's living conditions and quality of life. The development at the present stage is from the development of urgent and semi-interests to long-term interests and common interests, from the development of material resources to intangible resources or information resources (technology and knowledge).

The article "Analysis of the Implementation Effect of College Curriculum Ideological and Political under the Background of Ecological Sustainable Development" was retracted in 2023. Reasons: unreliable results or conclusions; concerns about the data; concerns about the peer review; concerns about the citations.

## 3. Research on Ideological and Political Education in Colleges and Universities under Ecological Sustainable Development

The analysis implementation effect course under the background of ecological sustainable development adopts the simulated ecological sustainable development model, constraints, and student course recommendation models. This model has a complete system, which can completely integrate a student's points of interest. The hobby of ideological and political courses is displayed, even if there is a little error, it is normal. After all, there are too many factors to be considered in the system. As long as the students make a little change, the results of the system will deviate; as long as the data is correct, then the final result has a high probability to meet the psychological expectations of the students, and the system also has a personal optimization function, which can be used to strengthen the results of the second calculation.

### 3.1. Establishment of an Optimal Configuration Model for Ecological Sustainable Development

Modelling methods can evaluate the evolution of the system against various design recommendations, and optimization methods are used to control the behavior of the system and develop strategies to understand the combination of modelling and optimization. The overall goal of system development is expressed through maximum overall benefit, generally in the following form:

(1) $$\begin{array}{c} Z=\max\left[F\left(X\right)\right]=\max\left\{S\left(X\right),J\left(X\right),H\left(X\right)\right\},G\left(X\right)\leq 0. \end{array}$$

The whole formula expresses the overall benefit in ecological sustainable development. *S* (*X*), *J* (*X*), and *H* (*X*), respectively, express the goals of social, economic, and environmental benefits. Analyzing the maximum interests, they can be regarded as the overall interests of the ecologically sustainable model. All of these three points will be studied later. *G* (*X*) is a limiting condition, which is to ensure that the system model can be well necessary constraint for its operation to continue, where *X* is the vector of solutions. *F* (*X*) is the total benefit function. *S* (*X*), *J* (*X*), and *H* (*X*) are the goals of social, economic, and environmental benefits, *G* (*X*) is a set of constraints, showing the ability of ecological environment resources, the ability to resist the environment, and the ability to carry land resources capacity and regional sublocal capacity.

The article "Analysis of the Implementation Effect of College Curriculum Ideological and Political under the Background of Ecological Sustainable Development" was retracted in 2023. Reasons: unreliable results or conclusions; concerns about the data; concerns about the peer review; concerns about the citations.

#### 3.1.1. Social Benefit

Social benefit is something that cannot be seen or touched, so it is not easy for us to make statistics and display it. We can transform the social benefit of ecological sustainable development into a specific thing, such as using water resources to measure social benefits. development, which can be a good reflection of the link between society and ecology:

(2) $$\begin{array}{c} \max S\left(X\right)=-\min\left[M_{J}^{K}-\sum_{c=1}^{L}X_{cj}^{k}\right]. \end{array}$$

Among them, these letters express the water consumption of the people in the *K* area and the total water storage capacity of the water source they use, and the following symbols almost all mean this.

#### 3.1.2. Economic benefits

Indirect economic benefits are brought about by the water supply of a region's ecological environment:

(3) $$\begin{array}{c} \max J\left(X\right)=\max\left[\sum_{i=1}^{I\left(k\right)}\left(b_{ij}^{k}-c_{ij}^{k}\right)+\sum_{C=1}^{L}\left(b_{cj}^{k}-c_{cj}^{k}\right)\right]. \end{array}$$

Formula (3) represents the economic benefits of water resources for the sustainable development of the ecological environment, which includes the economic coefficient of water resources and the clearly marked price of water resources provided. The proportion of the total reservoir and the cost of water consumption by each household can be optimized in the later stage. It ignores a function of saving water, and it should add a limit of forced water cutoff to avoid excessive water consumption and the depletion of the reservoir.

In, *b*_*ij*_^*k*^, *b*_*cj*_^*k*^ are the economic coefficient of water resources provided by two water source areas to *j* user units in *k* area, *c*_*ij*_^*k*^, *c*_*cj*_^*k*^. It is the cost of two water source regions to provide water resources to *j* user units in the *k* region. By enumerating these and calculating their maximum consumption and maximum water cost, the economic benefits of these two ecological environment regions can be simply obtained.

The article "Analysis of the Implementation Effect of College Curriculum Ideological and Political under the Background of Ecological Sustainable Development" was retracted in 2023. Reasons: unreliable results or conclusions; concerns about the data; concerns about the peer review; concerns about the citations.

#### 3.1.3. Ecological environmental benefits

The ecological environment generally includes water resources and land resources, and we will not discuss other bioclimatic resources. All the formulas listed are as follows:

(4) $$\begin{array}{c} \max H\left(X\right)=-\min\left[\sum_{k=1}^{k}\left(\sum_{i=1}^{I\left(K\right)}X_{ij}^{k}+\sum_{c=1}^{L}X_{cj}^{k}\right)\right]. \end{array}$$

*X*_*ij*_^*k*^indicates that area *k* meets the specific water demand of place *i* during a period of time; *X*_*cj*_^*k*^ means that the land resources in the *k* area meet the utilized land resources in the *j* area, and the two are combined to obtain the group maximum negative output value of the ecological environment.

### 3.2. Restrictions

Restrictions on water supply capacity of water resources and ecological environment are expressed as follows:

(5) $$\begin{array}{c} \left.\begin{array}{c} \sum_{j=1}^{J\left(K\right)}X_{cj}^{k}\leq M_{c}^{k}\\ \sum_{k=1}^{k}M_{c}^{k}\leq N_{c} \end{array}\right\}. \end{array}$$

Formula (5) has two meanings. The first is that the independent water source should be lower than the public water source, and the public water source should be smaller than the world's water reserves. This kind of restriction is realistic and can ensure the perfect operation of the system.

*Water Supply System Capacity Limitation*.

Public water source:

(6) $$\begin{array}{c} X_{cj}^{k}\leq Q_{C}. \end{array}$$

Independent water source:

(7) $$\begin{array}{c} X_{ij}^{k}\leq Q_{i}^{k}. \end{array}$$

*Q*_*C*_ is the maximum water supply capacity provided by the water source *C* that we can all use; *Q*_*i*_^*k*^ is the subregion of the *k* region with the largest water supply capacity.

The upper and lower limits of the water users need

(8) $$\begin{array}{c} M_{JL}^{K}\leq \sum_{i=1}^{I\left(k\right)}X_{ij}^{k}+\sum_{c=1}^{L}X_{cj}^{k}\leq M_{jH}^{k}. \end{array}$$

(4) Urban water discharge limit.

Minimum water discharge:

(9) $$\begin{array}{c} Z_{kg}^{t}\leq Z_{0}^{t}. \end{array}$$

Total limit:

(10) $$\begin{array}{c} \left[\sum_{k=1}^{K}\sum_{j=1}^{J\left(k\right)}0.01d_{j}^{k}p_{j}^{k}\left(\sum_{i=1}^{I\left(k\right)}X_{ij}^{k}+\sum_{c=1}^{L}X_{cj}^{k}\right)\right]\leq N_{0}. \end{array}$$

In, *d*_*j*_^*k*^ is the concentration of pollutants emitted by all users in the *k* area; *p*_*j*_^*k*^ is the discharge amount stipulated in my country; it is the total amount of pollutants allowed.

The article "Analysis of the Implementation Effect of College Curriculum Ideological and Political under the Background of Ecological Sustainable Development" was retracted in 2023. Reasons: unreliable results or conclusions; concerns about the data; concerns about the peer review; concerns about the citations.

Ecological environment constraints:

(11) $$\begin{array}{c} \sum_{k=1}^{K}\sum_{z=1}^{Z}X_{z}^{k}\leq S^{k}. \end{array}$$

Regional common development restrictions:

(12) $$\begin{array}{c} u=\sqrt{u_{A1}\left(\sigma_{1}\right)u_{A2}\left(\sigma_{2}\right)}\geq \overset{*}{u}, \end{array}$$

*u* is the actual adjustment; $\overset{*}{u}$ is the best adjustment; *A*_1_, *A*2 is an unclear subset of the connection between water use and regional economic development, and it is an unclear subset of the connection between local economic development and water environment quality improvement.

Nonnegative limit:

(13) $$\begin{array}{c} X_{ij}^{k}\cdot X_{cj}^{k}\geq 0. \end{array}$$

### 3.3. School Extracurricular Curriculum Proposal Model under Ecologically Sustainable Development

Traditional aggregation algorithms identify options by restricting connectivity and use attributes of existing useful fields to jointly predict and generate suggested assets. A complete process can bring the best results for your insurance. Due to the lack of some algorithms, the popular custom filter screen shows up in the early stages. When the following useful points are achieved for target users, strong data deletion cannot find strong data, resulting in poor real-time performance of the algorithm. When data shortages peak, new users can experience cold start issues, overloading the system. As long as the recipients of higher education and university science and policy are identified and aligned to some extent, screens of collaborative work are used to build high school concepts and models and encourage university policy recommendations.

#### 3.3.1. Collect Data to Establish Similarity Calculation

To avoid lack of raw data, a course that students liked in their minds in a variety of ways was found and classified according to different preferences, such as preliminary cold data collection; current noise and user errors, and data processing algorithms are used to filter out data noise. To limit the database to (0, 1), the database must be normalized. A common practice is to separate the different data with the highest value in that category. Vector methods are used to quantify similarity. According to the Euclidean–Read distance formula, if *X* and *Y* are two points in a multidimensional world, then the distance formulas of these two points are expressed as follows:

(14) $$\begin{array}{c} d\left(x,y\right)=\sqrt{{\left(\sum \left(x_{i}-y_{i}\right)\right)}^{2}}, \end{array}$$

(15) $$\begin{array}{c} V_{km}=C_{km}+a_{m}^{T}X_{k}. \end{array}$$

Among them, when *n* = 1, the calculated result is the distance between these two points. When *K* = 2, it represents the time required to walk the middle distance, but they are not perfect, we need to improve them:

(16) $$\begin{array}{c} \text{sim}\left(x,y\right)=\frac{1}{1}+d\left(x,y\right), \end{array}$$

(17) $$\begin{array}{c} {\text{VIF}}_{K}=\frac{1}{1-X_{X_{k}}^{2}}. \end{array}$$

Formula (16) represents the degree of liking of a course. It is reflected in the formula by the length of the distance. Formula (17) represents the time required to like this ideological and political course. With the addition of this formula, we can better observe the attitude changes of college students in the system and adjust the development in a timely manner and classify the students through the results obtained so as to better serve them and pick a course they like.

*x* and *y* indicate the degree of students' liking for a certain ideological and political course, and *K* still indicates the time it takes for them to complete the course.

The article "Analysis of the Implementation Effect of College Curriculum Ideological and Political under the Background of Ecological Sustainable Development" was retracted in 2023. Reasons: unreliable results or conclusions; concerns about the data; concerns about the peer review; concerns about the citations.

#### 3.3.2. Minimum Similarity Calculation of Neighbors

It limits the maximum value of students' political and ideological neighbors, and the distance to *K* is the neighborhood of the current point. Some students are adjacent to ideological and political courses, but there will not be much confusion and deviation in the selection of quantity; especially in personal matters, the advantages are obvious and the ability of students is improved. Neighborhood calculation in ideological and political direction:

(18) $$\begin{array}{c} F\left(z\right)=\exp\left[-\exp\left(-z\right)\right], \end{array}$$

(19) $$\begin{array}{c} p_{k}\left(m\right)=\sum_{q=1}^{Q}p_{k}\left(q\right)\times p_{klq}\left(m\right). \end{array}$$

#### 3.3.3. Calculation Recommendation

Based on the information of nearby students and nearby, a calculation recommendation mechanism is established, which aims at philosophers and political courses by taking “All students love political ideological course” as a vector. Following similar courses in the political ideal course, current students are predicted to show no interest based on the historical interest of the target students, and the consecutive, sequential order of the political ideal course is calculated in the form of a list of recommendations and predictions:

(20) $$\begin{array}{c} \text{CAIC}=-\ln\;L\left(a\right)+c\times \left(1+\ln\;K\right), \end{array}$$

(21) $$\begin{array}{c} \text{BIC}=-\ln\;L\left(a\right)+c\times \;\ln\;K. \end{array}$$

Not all students know what ideological and political courses they like, so we need to create formulas (20) and (21) for recommending ideological and political courses to help them choose courses. *A* and *k* are two ideological and political courses. For the overall database, if there are new ideological and political courses in the future, they will also be placed in these two. The calculation recommendation system is recommended for students in these two. If there is nothing they want at present, then when they like it, a similar course in the political ideals course is distributed to students based on the historical interests of the target students.

*a* and *k* are the overall databases of two courses; students choose favorite ideological courses among them; through these two formulas, relevant content for their chosen course is obtained.

The article "Analysis of the Implementation Effect of College Curriculum Ideological and Political under the Background of Ecological Sustainable Development" was retracted in 2023. Reasons: unreliable results or conclusions; concerns about the data; concerns about the peer review; concerns about the citations.

### 3.4. Optimization of Recommendation Model for Higher School Thought Courses

In view of the shortcomings of traditional collaborative filtering algorithms, the real-time recommendation model for ideological and political courses in colleges and universities is expanded, and the scope of application of the recommendation model for ideological and political courses in colleges and universities is expanded. It will become an advanced collaborative filtering algorithm for ideological and political courses in colleges and universities. Aiming at the actual needs of the in political and legal universities, an improved algorithm based on association grouping filtering is applied. By introducing a progressive curve based on user speed, the traditional grouping filtering algorithm has problems, such as low efficiency, poor adaptability, and exclusion.

#### 3.4.1. Introduce the Student History Hobby Mechanism

To overcome the problem of cold start of freshmen due to lack of reference materials, the historical association method is adopted to classify and link the historical interests of all students. A series of analogies are drawn with the combination of historical desires and similarities between ideology and political direction are calculated.

(22) $$\begin{array}{c} \text{sim}\left(i,j\right)=\frac{\sum_{u\in U}\left(R_{ui}-{\bar{R}}_{i}\right)\left(R_{uj}-{\bar{R}}_{j}\right)}{\sqrt{{\sum_{u\in U}\left(R_{ui}-{\bar{R}}_{i}\right)}^{2}}\sqrt{{\sum_{u\in U}\left(R_{uj}-{\bar{R}}_{j}\right)}^{2}}}. \end{array}$$

*U* is all students, *R*_*ui*_ and *R*_*uj*_, respectively, represent the data of students' historical interest in ideological and political courses, and ${\bar{R}}_{i}$ and ${\bar{R}}_{j}$ represent the students' average score evaluation of the course after taking the course.

#### 3.4.2. Introduce the Student's Forgetting Curve

Considering the changes of students' grade information over time, the historical fusion probability theorem is extended into a robust database that can continuously adapt to the rapid changes in students' real needs. It provides interest points for students in the new era and provides more concise, up-to-date, and personalized recommendations.. Due to the rapid dissemination of information about students' “level of interest,” students' choice of information results in a strong correlation between recommendation effectiveness and timing. By realizing the forgetting curve *R* = *e − t* and the comprehensive damping coefficient *s* (*u*, *v*, *i*) according to the actual situation of the student's area of interest and the optimization formula (22), the recommendation according to the recommendation time effect is synthesized, using the following formula:

(23) $$\begin{array}{c} s\left(u,v,i\right)=e^{-a}\frac{\left|t_{ui}-t_{vi}\right|}{t\max^{-t}t\min}. \end{array}$$

Formula (22) represents the student's history hobby formula, and formula (23) represents the student's forgetting formula. Both of these formulas are optimized for the recommendation model of college ideological and political courses and are both to better serve students. *Sustainable Development Ideological and Political Course*. With this student history, we can provide more thoughtful services to each student and also allow students who have attended the class to leave their opinions so that we can reform; introducing the forgetting curve can help us know the best of students. Memory points are sufficient, and students'course time can be arranged reasonably.

The article "Analysis of the Implementation Effect of College Curriculum Ideological and Political under the Background of Ecological Sustainable Development" was retracted in 2023. Reasons: unreliable results or conclusions; concerns about the data; concerns about the peer review; concerns about the citations.

In the appeal formula, *t*_*ui*_ and *t*_*vi*_ are the time required for student *u*, *v* to develop hobbies for an ideological and political course, |*t*_*ui*_ − *t*_*vi*_| is the hobby time gap between them, *t*max is the maximum time limit for students to generate hobbies, and *t*minrepresents the minimum time for students to generate hobbies. Equation (23) can be optimized to be more advanced:

(24) $$\begin{array}{c} sim\left(u,v\right)=\frac{\sum_{i\in l_{uv}}\left(R_{ui}-\overset{-}{R_{i}}\right)\left(R_{uj}-\overset{-}{R_{j}}\right)s\left(u,v,i\right)}{\sqrt{{\sum_{i\in l_{uv}}\left(R_{ui}-\overset{-}{R_{i}}\right)}^{2}}\sqrt{{\sum_{i\in l_{uv}}\left(R_{uj}-\overset{-}{R_{j}}\right)}^{2}}}. \end{array}$$

In the formula for calculating the similarity of student *u*, *v* political and ideological education choices, the decay factor in the forgetting curve is constrained by the student's hobby time and loss coefficient, indicating that the greater the time difference between student *u*, *v*, the more similar the students are. The performance will be reduced due to the reduction of the attenuation factor.

## 4. Experiment Analysis of Ecological Sustainable Development Integrated into College Curriculum Ideological and Political

### 4.1. The Necessity of Introducing Ecological Sustainable Development into College Curriculum

In a technical sense, “ecology” literally means “the violent evolutionary interaction between living things and organisms and between organisms and their natural environment.” Its essence is a strong and continuous connection between interconnected parts. Therefore, from an ecological point of view, we can also understand the harmonious interaction between organisms and the environment. The ecological system emphasizes the harmony and unity of organisms and the environment and the unity and balance of the system. It should be linked to the ideological and political education system in colleges and universities and requires unity and balance. Ideological and political education in colleges and universities reflects the relationship between teachers and students and their educational environment and reflects the core of “ecology.” Therefore, it is entirely possible to give full play to the professional benefits of high schools and to integrate the concept of ecological sustainable development into the ideological and political education of high schools and universities. Of course, this requires the strong support of my country. At present, the country with the best ecological sustainable development in the world is Japan. After it is proposed to integrate ecological sustainable development into the ideology and politics of college courses, my country's economic expenditure and Japan's economic expenditure are gradually decreasing.

The article "Analysis of the Implementation Effect of College Curriculum Ideological and Political under the Background of Ecological Sustainable Development" was retracted in 2023. Reasons: unreliable results or conclusions; concerns about the data; concerns about the peer review; concerns about the citations.

The investment in ecological sustainable development in my country and Japan is constantly increasing. My country has increased from 1.1 to 620 million yuan at the beginning, and Japan has increased from 5.4 to 690 million yuan. At the same time, my country's growth rate is significantly higher than that of Japan, the best ecological sustainable development country, but I believe that since our country has begun to pay attention to this issue, our country will surpass Japan to become the first in the near future.

According to the data in Figure 1 above, it can be seen that my country's ecologically sustainable economy is increasing rapidly every year, and the annual increase rate is faster than that of Japan, which is enough to prove my country's determination to change the ecological environment and sustainable economic development. It is believed that in the near future, my country will surpass Japan to become the first environmental protection country. Then, we selected some colleges and universities to investigate the attitudes of students. Through Figure 2, we got most of the students' support for this reform. After all, they are students in the new era, and most of them want to do meaningful thinking. They are also deeply aware of ecological protection awareness and sustainability.

The article "Analysis of the Implementation Effect of College Curriculum Ideological and Political under the Background of Ecological Sustainable Development" was retracted in 2023. Reasons: unreliable results or conclusions; concerns about the data; concerns about the peer review; concerns about the citations.

With the rapid development of the world's industry and the development and use of more energy, the problem of environmental pollution has become increasingly serious and diversified. People have gradually realized the threat and damage caused by environmental pollution to human beings and the natural environment, their awareness of environmental protection has been continuously enhanced, and they have realized the necessity and importance of ecological protection. The emergence and deepening of this awareness has further promoted the integration of ecological sustainable development into the development of ideological and political projects in college curricula. Among them, we focus on educating students on the current serious ecological and environmental problems, hoping that they can find better solutions in the future, as shown in Table 1.

### 4.2. Ideological and Political Content of College Courses

Ideological and political courses refer to the system in which schools use all ideological and political courses to carry out ideological and political education. There are several reasons for understanding and adopting this concept: First, ideological and political education is not a single course, but a system that includes the goals, content, methods, and methods of ideological and political education. Second, the “courses” referred to in ideology and politics refer to all ideological and political courses, including general courses, basic courses, specialized courses, and even secret courses without special learning forms. *Ideological and Political Course*. Therefore, the course is not part of the ideological and political course. Third, the field of ideological and political science teaching is ideological and political education, which is an important starting point for the practice of “three-dimensional education.” Fourth, ideology and procedure remain important concepts. As a new ideological and political concept, it is very important to promote the reform of ideological and political education; as an important concept of the curriculum, it gives the curriculum reform a broad position. It is shown in Table 2.

Systematically and effectively organizes its members to have specific ideology, political attitudes, and moral standards to shape their ideological and moral qualities. The main teachings include ecological sustainable development, college students' mental health, modern Chinese, mechanical design, and computer systems. We then applied predictive analytics to these to more quickly adapt to future changes, as shown in Figure 3.

The article "Analysis of the Implementation Effect of College Curriculum Ideological and Political under the Background of Ecological Sustainable Development" was retracted in 2023. Reasons: unreliable results or conclusions; concerns about the data; concerns about the peer review; concerns about the citations.

Among them, we can see that these are growing every year, and they have not stopped until 2016, which indirectly shows the importance of ideological and political education. But so many ideological and political courses will indirectly affect our own professional courses, and so on.

Figure 4 shows the student absorption rate after the course changes before and after the integration of ecological sustainable development and college ideological and political courses. Joining ideological and political courses has both advantages and disadvantages, such as ecological sustainable development and college students' mental health in the help of ideological and political courses In the next year, students like to listen to lectures more and more, and they absorb it better. On the contrary, their professional courses and advanced mathematics have declined.

### 4.3. The Situation after the Integration of Ecological Sustainable Development and Ideological and Political Courses in Colleges and Universities

After the integration of the two, the ecological environment in our country has been significantly reduced. By constantly giving students courses on ecological sustainable development, it subtly affects their thoughts and causes their actions to change. To drive the people around them, after a period of time, we investigated some data to analyse their teaching mode and ecological environment, as shown in Table 3 and Table 4.

It is necessary to carry out this reform through investigation and analysis. Through the data, it can be clearly found that the ecological environment has become better, and the living environment of the students has become better and better. After introducing a system that combines historical priorities and a rate-of-change-based system, we compared the model proposal's real impact on the curriculum of political thought schools, confirming that it is general and objective.

From the above data in Figure 5, it can be seen that the more times the ecological sustainable development algorithm is run, the higher its overall stability, so it is very suitable to use this algorithm. Finally, if you want to make college students effective, you can start from the following points in Figure 6:

After completing the ideological and political courses of ecological sustainable development, college students have produced many good changes in their actions. In terms of environmental protection, they learned to use less disposable chopsticks, know what kind of garbage to throw in which trash can when throwing garbage, and so on. In school, they learned to save food and turn off taps in time. At home, they would appeal to parents, acting together for ecological and economic sustainability.

The article "Analysis of the Implementation Effect of College Curriculum Ideological and Political under the Background of Ecological Sustainable Development" was retracted in 2023. Reasons: unreliable results or conclusions; concerns about the data; concerns about the peer review; concerns about the citations.

It can be seen that all these points have increased in this year, which shows that the implementation effect analysis of college curriculum ideology and politics under the background of ecological sustainable development is very good, and it can continue to develop in the future.

## 5. Conclusion

The theme is the analysis of the implementation effect of college curriculum ideology and politics under the background of ecological sustainable development, which discusses the definition of ecological sustainable development, the principles of ecological sustainable development, and the significance of developing ecological sustainable development. Design and experiment the ideological and political research model of colleges and universities under the ecological sustainable development, and design experiments so that many students can recommend an ideological and political course for them to learn when they hesitate in colleges and universities, although ecological issues are now integrated into college ideological and political courses. There are many problems, but due to the development of the form and the times, it will be solved sooner or later. Now we should seize the opportunity to improve the usefulness of this theme, strengthen the ideological and political development of the future ecological sustainable development of colleges and universities, and make up for it. Its shortcomings pave the way for its rapid development in the future.

## Figures and Tables

**Figure 1:** Comparison of economic spending between China and Japan.

**Figure 2:** Survey of students.

**Figure 3:** Ideological and political courses.

**Figure 4:** Absorption rate of students before and after.

**Figure 5:** Comparison of the accuracy of the two recommendations before and after optimization.

**Figure 6:** Analysis of the actual effect.

**Table 1:** Teaching content.

Learning content	Solution	Teaching percentage
Water pollution problem	Strictly control urban sewage discharge	25%
Air pollution problem	Particulate pollutant purification technology	25%
Solid waste disposal issues	More recycling	15%
Noise and radioactive pollution issues	Take strict protective measures	20%
Comprehensive prevention of pollution	Reasonable planning and layout of resources	15%

**Table 2:** Ideological and political analysis.

Ideological and political analysis	Content	Proportion
The essence of ideological and political courses	Realizing ideological and political collaborative education with curriculum as the carrier	25.20%
Characteristics of ideological and political courses	Extensiveness, occultity, and diversity	30.20%
Difficulties of ideological and political courses	The integration of ideology and politics and students and the contradiction of the system	15.00%
Ideological and political course innovation	Using the Internet as a technology to strengthen ecological sustainable development	34%

The article "Analysis of the Implementation Effect of College Curriculum Ideological and Political under the Background of Ecological Sustainable Development" was retracted in 2023. Reasons: unreliable results or conclusions; concerns about the data; concerns about the peer review; concerns about the citations.

**Table 3:** Analysis of fusion mode.

Three phases	Content
Before class	Online preparation based on web platform
After class	Offline teaching based on traditional classroom
After class	Extracurricular supplements based on practical activities

**Table 4:** Pollution changes.

Pollution source	Changes	Reason
Air pollution	25%–20%	Businesses take advantage of clean combustion sources
Soil erosion	18%–15%	Students save water every day
Greening reduction	8%–7%	Students are very young using disposable chopsticks
Acid rain formation	3%–2.5%	Less frequent use of coal

## Data Availability

The experimental data used to support the findings of this study are available from the corresponding author upon request.
